# How Technological Innovation Affect China's Pharmaceutical Smart Manufacturing Industrial Upgrading

**DOI:** 10.1155/2021/3342153

**Published:** 2021-11-26

**Authors:** Su Wang, Yuwen Chen

**Affiliations:** School of Business Administration, Shenyang Pharmaceutical University, Shenyang 110016, China

## Abstract

In recent years, a new generation of information technology has provided sufficient technical support for the smart manufacturing industry. In order to promote the upgrading of China's pharmaceutical smart manufacturing industry, the direction of industrial upgrading and transformation will be discussed from the perspective of technological innovation. According to the input and output data of technological innovation in China's pharmaceutical manufacturing industry from 2007 to 2019, the DEA method is used to analyze the allocation of innovative resources in China's pharmaceutical manufacturing industry in recent years. The study found that the efficiency of technological innovation in China's pharmaceutical manufacturing industry fluctuated greatly from 2007 to 2019, with a low overall level and varying degrees of wasted resources. On this basis, an in-depth analysis of the system architecture of the pharmaceutical smart manufacturing industry under the Industry 4.0 environment was performed. Finally, four paths for the digital transformation of China's pharmaceutical manufacturing industry are proposed. Chinese pharmaceutical manufacturing companies need to use new technologies to carry out comprehensive intelligent upgrading and digital transformation to improve innovation efficiency.

## 1. Introduction

China's smart manufacturing industry has made some achievements in recent years. Smart manufacturing exerts a profound influence on the pharmaceutical industry, leading to the following three development trends [1–3]. The first is improving the intelligence and information levels of the pharmaceutical industry and popularizing manufacturing execution systems to the production processes, thereby achieving the whole-process monitoring and management of drug quality. The second is innovation of the production techniques and enhancing the applications of computer-aided drug design, 3D printing, and virtual reality during research and development (R&D). The third is increasing industry concentration, shifting the market structure of the pharmaceutical industry based on industrial integration, and promoting the pharmaceutical industry to the international market. Smart manufacturing in China's pharmaceutical industry is at the primary stage; characteristics of the pharmaceutical industry put forward loads of special needs on smart manufacturing. Competitive situations in China's manufacturing industry have become increasingly fierce, and production costs and labor costs have increased accordingly. Manufacturing corporates, including pharmaceutical corporates, have begun to use new technologies to improve production efficiency and strengthen product innovation and management capabilities, gaining competitive advantages [4]. Hence, the smart upgrade of the pharmaceutical manufacturing industry is crucial to the industry's long-term development in this context.

As the pharmaceutical industry becomes smarter in pharmaceutical production, promoting the smart development of pharmaceutical manufacturing corporates through pharmaceutical equipment and helping corporates transform from automated production to smart production has become the road to the smart development of pharmaceutical manufacturing corporates [5, 6]. As a typical innovation-driven and technology-intensive industry, pharmaceutical manufacturing is characterized by high thresholds and high risks. Hence, it is difficult for a corporate to depend on its accumulation to break through the dilemma between R&D and continuous growth [7]. Innovation is the first driving force for development, and the pharmaceutical manufacturing industry is a critical carrier that can best embody technological competitiveness. Hence, technological innovation has become a decisive factor in the competitiveness of pharmaceutical manufacturing corporates. Continuous optimization and innovation of enterprise technology are the keys to ensuring the quality of medicine and improving efficiency.

Some factors restrict the current innovation and development of the pharmaceutical manufacturing industry in China, and the smart agglomeration effect must be expanded further. This paper deeply analyzes the current technological innovation input and output of China's pharmaceutical manufacturing industry. It evaluates the technological innovation efficiency of China's pharmaceutical manufacturing industry from 2007 to 2019 and clarifies the allocation of innovative resources in China's pharmaceutical manufacturing industry in recent years. Based on the evaluation results, combined with the development needs of the pharmaceutical manufacturing industry, we clarify the necessity of technological innovation and intelligent upgrading of China's pharmaceutical manufacturing enterprises and propose specific transformation paths. The innovation point is to help China's pharmaceutical smart manufacturing industry achieve industrial upgrading through theoretical analysis and empirical research from the perspective of accelerating technological innovation and improving the efficiency of technological innovation in the pharmaceutical industry.

## 2. Evaluation of Technological Innovation Efficiency in China's Pharmaceutical Manufacturing Industry

### 2.1. Input and Output of China's Pharmaceutical Manufacturing Industry Technological Innovation

There are multiple choices for corporate R&D innovation models, which should be comprehensively considered based on the specific R&D time, personnel, and R&D difficulty of the corporates. Corporate R&D innovation is a process of trial and error. According to different R&D subjects, R&D innovation modes can be divided into independent innovation, cooperative innovation, and imitative innovation. Independent innovation means that corporates develop products depending on their technical capabilities and realize the productization of R&D results on this basis, thereby gaining market recognition. Cooperative innovation is an innovative organization formed by cooperation among multiple corporates and research institutions [8–10]. Some large-scale and complex innovation activities often require cooperative innovation among multiple units, giving full play to their respective advantages, achieving complementary resources, and providing the possibility of successful innovation. Imitative innovation introduces new technologies through legal means under the influence of other corporates' pioneering innovations and improves the original technology system [11, 12]. Usually, before imitative innovation, high-quality imitation is performed first. Then, some entry points for improvement can be found.

Innovation activities of the pharmaceutical manufacturing industry are divided into two stages: the input stage and the output stage. The technological innovation of pharmaceutical manufacturing corporates requires the support of inputs such as funds and personnel. R&D expenditure and personnel input directly manifest the importance of a pharmaceutical manufacturing corporate to R&D, which is also the power source for future development. Using capital and personnel inputs to transform into knowledge output efficiently and economic output is undoubtedly the industry's lifeblood and the driving factor for developing pharmaceutical manufacturing enterprises [13]. The R&D internal expenditure and R&D external expenditure of China's pharmaceutical manufacturing industry during 2012–2019 are illustrated in Figure 1; the new products development expenditure and full-time equivalent on R&D personnel of China's pharmaceutical manufacturing industry during 2012–2019 are presented in Figure 2 (data source: China National Bureau of Statistics).

Figure 1 shows that the total internal expenditure of R&D and external expenditure of R&D in China's pharmaceutical manufacturing industry showed a year-on-year growth trend from 2012 to 2019. Internal expenditure of R&D increased from 283.31 hundred million yuan in 2012 to 609.56 hundred million yuan in 2019, an increase of 2.15 times and an average annual growth rate of 11.57%. External expenditure of R&D increased from 33.86 hundred million yuan in 2012 to 110.62 hundred million yuan in 2019, an increase of 3.27 times, with an average annual growth rate of 18.43%, with the most significant increase in 2018. It shows that, in recent years, Chinese pharmaceutical manufacturing enterprises have attached great importance to independent innovation and cooperative innovation activities and have continuously increased capital investment to ensure the innovative development of enterprises.

Figure 2 shows that the total expenditure on new products development in China's pharmaceutical manufacturing industry has increased year-on-year from 308.23 hundred million yuan in 2012 to 732.52 hundred million yuan in 2019, an increase of 2.38 times, with an average annual growth rate of 13.16%. It shows that China's pharmaceutical manufacturing industry has paid more attention to new products development and design investment in recent years, which is an essential guarantee for improving industrial innovation. The full-time equivalent on R&D personnel in China's pharmaceutical manufacturing industry showed a fluctuating growth trend from 2012 to 2019. It increased significantly from 2012 to 2014 and reached the highest investment value in recent years by 2014. In 2015, it decreased for the first time, from 133900 man-years in 2014 to 128600 man-years in 2015. From 2016 to 2019, there was a volatile downward trend. In 2019, the full-time equivalent on R&D personnel reached 122700 man-years.

Pharmaceutical manufacturing is a particular industry, and its innovation results must be tested through clinical trials, requiring an extended period. Products and patents owned by a corporate can serve as an essential indicator of its technological innovation output. The new products sales revenue and patent applications of China's pharmaceutical manufacturing industry during 2012–2019 are demonstrated in Figure 3.

Figure 3 shows that the sales revenue of new products in China's pharmaceutical manufacturing industry has increased year-on-year from 2928.6 hundred million yuan in 2012 to 6673.46 hundred million yuan in 2019, an increase of 2.28 times, with an average annual growth rate of 12.49%. It shows that, with the continuous improvement of the R&D input of China's pharmaceutical manufacturing industry, the economic benefits have gradually improved. The number of patent applications in China's pharmaceutical manufacturing industry showed a fluctuating growth trend, from 14976 in 2012 to 23400 in 2019, an increase of 1.56 times. There was only a short-term downward trend in 2015 and continued growth in the rest of the year. It shows that while China's pharmaceutical manufacturing industry attaches importance to drug R&D and innovation, its awareness of patent protection is also increasing. Under the combined action of demand growth, technological innovation, policy encouragement, talent gathering, and capital input, China's pharmaceutical manufacturing industry will be in a golden development period for some time in the future, showing a pattern of scale expansion, innovation upgrading, and competition differentiation [14, 15].

### 2.2. Method

This paper uses the data envelopment analysis (DEA) method proposed by Charnes et al. [16] to evaluate the technological innovation efficiency of China's pharmaceutical manufacturing industry. The evaluation methods of innovation efficiency mainly include the parametric method and nonparametric method. Since the allocation of innovative resources is a complex system with multiple inputs and multiple outputs, compared with the parametric method, the nonparametric method does not need to estimate the parameters in advance, which is more in line with the multiple optimization criteria. DEA is representative of nonparametric methods, and it is also an effective method commonly used to evaluate the efficiency of technological innovation. It does not require model parameters, only multiple input and output data to calculate the effective frontier and then calculate the distance between each decision-making unit (DMU) and the effective frontier, thereby evaluating the relative effectiveness of each DMU.

DEA method mainly includes CCR and BBC model. The CCR model can calculate the relative efficiency under constant returns to scale. The BBC model is an improvement based on the CCR model, which calculates relative efficiency under variable returns to scale. This paper selected the DEA-BBC model with variable returns to scale to evaluate the relative efficiency of technological innovation in China's pharmaceutical manufacturing industry over 13 years (2007–2019). For any DMU, the BBC model [17] under input orientation is as follows:

(1) $$\begin{array}{c} \min,\left[\theta -\varepsilon \left(\sum_{i=1}^{m}s^{-}+\sum_{r=1}^{s}s^{+}\right)\right],\\ s\mathrm{.t}..\;\left\{\begin{array}{c} \sum_{j=1}^{n}\lambda_{j}x_{ij}+s^{-}=\theta x_{i0}\\ \sum_{j=1}^{n}\lambda_{j}y_{rj}+s^{+}=y_{r0}\\ \sum_{j=1}^{n}\lambda_{j}=1\\ \lambda_{j}\geq 0,s^{+}\geq 0,s^{-}\geq 0 \end{array}.\right) \end{array}$$

In model (1), *j*=1,2,…, *n*; *i*=1,2,…, *m*; *r*=1,2,…, *s*. *n* is the number of DMUs (years in our case); *m* and *s* are the number of input and output variables. *x*_*ij*_ and *y*_*rj*_ are input and output variables. *s*^−^ and *s*^+^ are the slack variables of input and output. *θ* is the effective value; *ε* is the non-Archimedean infinitesimal. When *θ* is 1, it means that the DMU is relatively efficiency, and when it is less than 1, it is inefficiency.

### 2.3. Research Sample

Technological innovation is a multi-input and multi-output economic process. In the process of efficiency evaluation, choosing appropriate input and output indicators is crucial to the effectiveness of the evaluation results. The innovation input of the pharmaceutical manufacturing industry mainly includes capital and personnel input. Four input indicators are selected for the efficiency model: internal expenditure of R&D, external expenditure of R&D, new products development expenditure, and full-time equivalent on R&D personnel. The internal expenditure of R&D refers to the expenditure of a company to independently research and develop a specific technology, which promotes the internal generation of new knowledge and can promote various innovative activities [18]. External R&D expenditures are expenditures in the process of joint R&D activities carried out by enterprises and partners. This model is conducive to speeding up the R&D process of new technologies and knowledge [19]. New product development expenditures reflect the expenditures in a series of processes, including product, process design, production, and market expansion. The full-time equivalent on R&D personnel is a more accurate reflection of the workforce input in technological innovation. The outputs included in the analysis are as follows: sales revenue of new products and number of patent applications, reflecting the economic output and knowledge output of technological innovation activities. The definition of input and output variables is shown in Table 1.

The data used for efficiency analysis comes from the “China High-Tech Industry Statistical Yearbook” and “China Science and Technology Statistical Yearbook.” Given the availability of data, this paper selects the relevant data of China's pharmaceutical manufacturing industry from 2005 to 2019 and uses DEAP2.1 software to analyze the efficiency of technological innovation. Due to the hysteresis of innovation activities, the year's input cannot be converted into output immediately. Therefore, this paper draws on Furman's method and sets the lag period to two years [20]. The input indicator is the 2005–2017 data, and the output indicator is the 2007–2019 data. Each year is regarded as the DMUs, and the relevant data is shown in Table 2.

## 3. Results and Discussion

### 3.1. Correlation Tests of Innovation Indicators

Before measuring the technological innovation efficiency of China's pharmaceutical manufacturing industry, the Pearson correlation test should be performed on the input and output indicators. The results are shown in Table 3. The test results show that the correlation coefficient between innovation input and output indicators is more significant than 0.8 at the level of 1%, which has a strong correlation. Therefore, the innovation input and output indicators selected in this paper are more reasonable, further measuring and analyzing technological innovation efficiency.

### 3.2. Technological Innovation Efficiency of China's Pharmaceutical Manufacturing Industry

Table 4 shows the technological innovation efficiency score of China's pharmaceutical manufacturing industry from 2007 to 2019. One indicates the year as efficient and anything less as inefficient. Variation trends of efficiency are shown in Figure 4.

Dynamic and longitudinal analysis of technological innovation efficiency can understand the specific technological innovation resource allocation situations in China's pharmaceutical manufacturing industry. During 2007–2019, the overall technological innovation efficiency of China's pharmaceutical manufacturing industry fluctuated greatly and was inefficient, with an efficiency average of 0.832. Only three years, 2009, 2012, and 2019, were efficient over the 13-year period. Technological innovation resource allocation was reasonable in 2012, 2013, and 2019. In contrast, situations were terrible in 2007, 2011, 2013, and 2015, and resources were wasted seriously. By taking the mean value during 2007–2019 as the baseline, the technological innovation efficiency in China's pharmaceutical manufacturing industry has increased by 17.8% in 2019. By taking 2007 as the baseline, the technological innovation efficiency in 2019 has increased by 27.2%.

## 4. Transformation and Smart Upgrading of China's Pharmaceutical Manufacturing Industry

### 4.1. Pharmaceutical Smart Manufacturing System Architecture

Combining new technology and advanced manufacturing has become an important strategic direction for various industries with the rapid development of a new generation of information technology. As one of the high-tech industries, the pharmaceutical manufacturing industry has gradually improved its intelligence level to maintain competitiveness. The automation and information construction level of China's pharmaceutical manufacturing industry is relatively low compared with other industries. After evaluating the innovation efficiency of China's pharmaceutical manufacturing industry, the overall innovation efficiency level was low, and it was in a low-efficiency state in most years. Strategies such as Industry 4.0 and the Industrial Internet have put pharmaceutical manufacturing corporates in the midst of information transformation. Pursuing the corporate sustainable development model, enhancing the corporate information application and management levels, and achieving smart manufacturing are crucial subjects of the pharmaceutical manufacturing industry [21]. Pharmaceutical smart manufacturing and Pharmaceutical Industry 4.0 can monitor all the pharmaceutical manufacturing and circulation processes in real-time online, effectively improving R&D and production efficiency. Moreover, data can be generated and read automatically and stored in the cloud directly, with zero delays and no blind spots [22]. A complete pharmaceutical smart manufacturing system comprises four layers: the equipment layer, the control layer, the business management layer, and the operating management layer. The system architecture is demonstrated in Figure 5 [23–25].

The equipment layer is usually composed of single hardware such as automated operating equipment, meters, and sensors. It is responsible for specific production tasks, providing underlying data support for production process control. The equipment layer can configure equipment that meets the requirements according to the corporate business scope and management needs. The control layer docks with the equipment layer, which is responsible for collecting and integrating data about the equipment layer. Hence, it is the basis of information management for smart manufacturing [26]. Corporates can achieve preliminary visual management through data integration in the control layer and further optimize the digital function structure and information flow structure. The business management layer can achieve the integrated application of business management in the smart manufacturing industry. People, machines, and materials can be fully integrated by optimizing and reconstructing the business management layer. The business management layer is connected to the operating management layer. As the transmitter of corporate management decisions, it is a key link to constructing the smart manufacturing system. The operating management layer straddles other systems and runs through the entire process of research, development, production, quality control, and logistics. It is the core for pharmaceutical manufacturing corporates to meet the management requirements of global optimization. An important prerequisite for the operating management layer to play the role of intelligent decision-making is the interconnection among the business management layer, the control layer, and the equipment layer. Important information can be visually displayed through data analysis to assist decision-making. The software system in the operating management layer helps the pharmaceutical manufacturing corporate realize top-down centralized management.

### 4.2. Smart Digital Transformation Path for China's Pharmaceutical Manufacturing Industry

In the broad concept of medical and health, pharmaceutical is the backbone of the medical and health ecosystem. The pharmaceutical industry must follow the trend, fit the trend of digital development, actively seek new mutations, and better contribute to the advancement of the medical and health industry. Digitization is the foundation of smart manufacturing. Regarding the current pharmaceutical market development, the pharmaceutical industry digitalization has an excellent market foundation [27]. In 2018, the scale of China's digital economy reached 31.3 trillion Chinese yuan; during the same period, China's Gross Domestic Product (GDP) reached 91.9 trillion Chinese yuan. Hence, China's digital economy accounted for 34.8% of its GDP in 2018. Calculated on a comparable basis, the digital economy scale achieves a nominal growth of 20.9%, and its occupation increases by 1.9%. The pharmaceutical industry maintains a relatively high industry growth rate, with a market growth rate of about 10%. However, the overall digitalization degree is relatively low.  Figure 6 shows the market scale and digital transformation trend of China's pharmaceutical. Therefore, the long-term high-speed industry growth rate and the low digitization at this stage are both an opportunity and a challenge for the pharmaceutical industry digitization.

In the context of structural adjustment and overall upgrading of the pharmaceutical industry, pharmaceutical companies have gradually realized the importance of building a digital system. The current application of digital technology in pharmaceutical companies has four paths from a value perspective. The first path is enabling scientific research. New drug research and development is the beginning of the entire drug life cycle. Through digital empowerment, the storage, integration, feedback, management, and in-depth mining of a large number of preclinical and clinical trial research data can reduce R&D costs, speed up the development process, and improve the success rate of research and development [28]. The second path is improving the quality of medicines. Compared with other industries, the pharmaceutical industry has stricter requirements on product quality, and the stability of drug quality is the foundation of its market value. The application of quality digitization is conducive to ensuring the quality of drugs and is also the key to the entire life cycle of drugs. It is mainly used in process design, production process monitoring, and drug batch evaluation [29]. Through quality digital technology, it is possible to track and monitor whether the whole-process meets the quality specifications, minimize the influence of human factors, strengthen the standardization of the process, and continuously improve the quality of medicines. The third path is optimizing the production process. The use of digital technology can monitor the status and potential risks of production equipment in real-time, reduce nonproduction use time, and effectively avoid risks. It can also make scientific decisions based on visual data analysis for production scheduling and storage of production materials to improve production efficiency. The fourth path is reorganizing business operations. Standard reports and accumulations produced by digital technology can provide valuable data for business operators and improve business efficiency. The massive data analysis provides scientific and effective decision-making for operation management personnel based on indicators such as cost, workforce, and procurement. It also feeds back information such as business performance and risks to business managers in real-time, enhances business decision-making capabilities, and optimizes business development directions and models [30].

## 5. Conclusion and Future Research

### 5.1. Conclusion

Pharmaceutical manufacturing is vital to people's health, which has become a key strategic industry in China. The rapid development of the new generation of intelligent manufacturing technology has become a key factor driving the sustainable development of the pharmaceutical manufacturing industry. This paper comprehensively analyzes China's pharmaceutical manufacturing industry's technological innovation status and efficiency and provides a basis for intelligent industrial upgrading. According to the data on technological innovation input and output of China's pharmaceutical manufacturing industry from 2007 to 2019, the specific allocation of innovation resources is dynamically analyzed. From 2007 to 2019, the overall technological innovation efficiency of China's pharmaceutical manufacturing industry was low, with an average efficiency of 0.832. In 2009, 2012, and 2019, the allocation of innovation resources was reasonable, and the other years had varying degrees of waste of innovation resources. Based on 2007, the technological innovation efficiency of China's pharmaceutical manufacturing industry increased by 27.2% in 2019. Finally, four paths for the digital transformation of Chinese pharmaceutical companies are proposed. In response to the current situation, Chinese pharmaceutical manufacturing companies should actively change business philosophy, focus on the full use of new technologies, comprehensively carry out intelligent upgrades and digital transformations, and further improve innovation efficiency. The research results are of great value in clarifying the current state of technological innovation in China's pharmaceutical manufacturing industry and the direction of upgrading the pharmaceutical smart manufacturing industry.

### 5.2. Future Research

In the context of the rapid development of a new generation of information technology, the pharmaceutical manufacturing industry has huge technological innovation potential. The pharmaceutical smart manufacturing industry can reduce R&D costs, ensure the quality of medicines, and improve efficiency. After evaluating the innovation efficiency of China's pharmaceutical manufacturing industry, it was found that the efficiency of resource allocation is low. It proposes the direction of industrial upgrading and digital transformation from a theoretical level and provides new ideas for the intelligent upgrade of the pharmaceutical manufacturing industry. However, the impact of new technologies on the intelligent upgrade of the pharmaceutical manufacturing industry has not yet been quantitatively studied. Therefore, in future research, empirical analysis can be carried out by collecting indicator data to reflect the level of new technologies and intelligent upgrades to make the impact mechanism clearer.

## Figures and Tables

**Figure 1:** R&D internal expenditure and R&D external expenditure of China's pharmaceutical manufacturing industry during 2012–2019.

**Figure 2:** New products development expenditure and full-time equivalent on R&D personnel of China's pharmaceutical manufacturing industry during 2012–2019.

**Figure 3:** New products sales revenue and patent applications of China's pharmaceutical manufacturing industry during 2012–2019.

**Figure 4:** Variation trends of technological innovation efficiency in China's pharmaceutical manufacturing industry during 2007–2019.

**Figure 5:** Smart manufacturing system architecture for pharmaceutical manufacturing corporates.

**Figure 6:** Market size and digital transformation trend of China's pharmaceutical (data source: Frost & Sullivan). (a) The scale of China's pharmaceutical market. (b) Digital transformation of pharmaceutical market.

**Table 1:** Definition of input and output variables.

Variable	Role	Definition
Internal expenditure of R&D (100 million yuan)	Input (*x*1)	The actual expenditure of the enterprise for internal R&D activities (basic research, applied research, and experimental development)
External expenditure of R&D (100 million yuan)	Input (*x*2)	Funds paid by enterprises to cooperative organizations include expenditures for acquiring technology from domestic scientific research institutes and domestic and foreign enterprises
New products development expenditure (100 million yuan)	Input (*x*3)	The internal expenditures for enterprises' scientific and technological activities are used for the R&D of new products
Full-time equivalent on R&D personnel (man-year)	Input (*x*4)	The number of full-time personnel plus part-time personnel is converted into the total number of full-time personnel according to the workload
Sales revenue of new products (100 million yuan)	Output (*y*1)	The sales revenue realized by the enterprise selling new products
Number of patent applications (piece)	Output (*y*2)	The number of patents applied for by enterprises, including invention patents, utility model patents, and design patents

**Table 2:** Efficiency data.

DMUs	*x*1	*x*2	*x*3	*x*4	*y*1	*y*2
1	39.95	15.65	44.77	19584	712.69	3056
2	52.59	15.52	55.76	25391	948.91	3917
3	65.88	18.22	73.94	30778	1592.46	8601
4	79.09	18.04	87.19	40192	1675.53	5767
5	134.54	19.96	155.06	70065	2317.04	11115
6	122.63	17.72	131.40	55234	2928.60	14976
7	211.25	45.29	233.07	93467	3606.17	17124
8	283.31	33.86	308.23	106684	4301.84	19354
9	347.66	40.82	364.50	123200	4736.27	16020
10	390.32	48.28	407.93	133902	5422.75	17785
11	441.46	52.86	427.95	128589	5713.25	19878
12	488.47	60.05	497.88	130570	6367.04	21698
13	534.18	68.86	588.60	121517	6673.46	23400

**Table 3:** Correlation test results of innovation indicators.

Variable	Internal expenditure of R&D	External expenditure of R&D	New products development expenditure	Full-time equivalent on R&D personnel
Sales revenue of new products	0.987^*∗∗∗*^	0.949^*∗∗∗*^	0.985^*∗∗∗*^	0.959^*∗∗∗*^
Number of patent applications	0.906^*∗∗∗*^	0.881^*∗∗∗*^	0.912^*∗∗∗*^	0.917^*∗∗∗*^

^*∗∗∗*^ *p* < 0.01.

**Table 4:** Efficiency score.

Years	Efficiency
2007	0.738
2008	0.764
2009	1.000
2010	0.881
2011	0.721
2012	1.000
2013	0.727
2014	0.769
2015	0.724
2016	0.759
2017	0.827
2018	0.901
2019	1.000
Mean	0.832

## Data Availability

The data used to support the findings of this study are included within the article.
